# A Variable Radius Side Window Direct SLAM Method Based on Semantic Information

**DOI:** 10.1155/2022/4075910

**Published:** 2022-08-22

**Authors:** Yan Chen, Jianjun Ni, Emmanuel Mutabazi, Weidong Cao, Simon X. Yang

**Affiliations:** ^1^College of Internet of Things Engineering, Hohai University, Changzhou 213022, China; ^2^Jiangsu Key Laboratory of Power Transmission & Distribution Equipment Technology, Hohai University, Changzhou 213022, China; ^3^Advanced Robotics and Intelligent Systems (ARIS) Laboratory, School of Engineering, University of Guelph, Guelph, ON, Canada

## Abstract

Simultaneous Localization and Mapping (SLAM) is a challenging and key issue in the mobile robotic fields. In terms of the visual SLAM problem, the direct methods are more suitable for more expansive scenes with many repetitive features or less texture in contrast with the feature-based methods. However, the robustness of the direct methods is weaker than that of the feature-based methods. To deal with this problem, an improved direct sparse odometry with loop closure (LDSO) is proposed, where the performance of the SLAM system under the influence of different imaging disturbances of the camera is focused on. In the proposed method, a method based on the side window strategy is proposed for preprocessing the input images with a multilayer stacked pixel blender. Then, a variable radius side window strategy based on semantic information is proposed to reduce the weight of selected points on semistatic objects, which can reduce the computation and improve the accuracy of the SLAM system based on the direct method. Various experiments are conducted on the KITTI dataset and TUM RGB-D dataset to test the performance of the proposed method under different camera imaging disturbances. The quantitative and qualitative evaluations show that the proposed method has better robustness than the state-of-the-art direct methods in the literature. Finally, a real-world experiment is conducted, and the results prove the effectiveness of the proposed method.

## 1. Introduction

Simultaneous Localization and Mapping (SLAM) plays essential roles in robotic and other related fields [1–3]. In the robotic field, SLAM systems are used to solve the problem of robots about where they are. Based on the acquisition of its pose and surrounding environment, a robot can further solve where to go or what to do [4].

Many kinds of sensors are used in SLAM systems, such as LiDAR, camera, and inertial measurement unit [5, 6]. Commonly, SLAM algorithms are divided into laser SLAM and visual SLAM according to the sensor used [7, 8]. Due to the low cost of the camera, the large amount of information it carries, and the ease of use, visual SLAM has become more popular among researchers in recent years. Visual SLAM usually uses monocular cameras, binocular cameras, or RGB-D cameras to obtain environmental information. Compared with other types of cameras, the monocular camera is cheap and common. In addition, there are the most abundant data sources of the monocular camera. So the monocular SLAM plays an important role in the visual SLAM field and has been widely studied and applied [9, 10]. However, the monocular SLAM can obtain only image information without scale information, so it is more dependent on the quality of the image. Therefore, how to improve the robustness of monocular SLAM under different disturbances is a very challenging and important task in this field [11, 12].

There are three main implementation schemes in visual SLAM, namely feature-based method, direct method, and semidirect method. The feature-based method finds feature points, matches them, calculates the pose, and constructs a map through geometric relations. The most commonly used methods for feature extraction are Scale Invariant Feature Transform (SIFT) [13], Speeded Up Robust Features (SURF) [14], and Oriented Fast and Rotated BRIEF (ORB) [15]. ORB is one of the best methods, which improves the speed and accuracy of FAST [16], and uses BRIEF [17] for the efficient computation of features. Accordingly, ORB-SLAM is currently the most popular visual SLAM solution [18, 19].

Unlike the feature-based method, the direct approach does not rely on the one-to-one matching of points. It optimizes the interframe pose by extracting pixels with apparent gradients and minimizing the photometric error function of the pixels, such as the large-scale direct monocular SLAM (LSD-SLAM) [20] and the direct sparse odometry (DSO) [21]. The semidirect method, such as the semidirect visual odometry (SVO) [22], uses a similar structure to the feature-based method and combines the tracking of the direct method and the motion optimization of the feature-based method. The feature-based method and the semidirect method both rely on low-level geometric feature extractors with high repeatability. They are not suitable for surfaces with many repetitive features or less texture. In contrast, the direct method can be used in a broader range of scenarios. In this paper, we focus on direct method solutions for the monocular SLAM. The main purpose of this paper is to improve the robustness of the direct methods under different disturbances.

The robustness of the direct method-based SLAM system is challenged by photometric calibration, dynamic objects, rolling shutter effect, camera imaging disturbances, and so on [23]. There have been many excellent works to improve the robustness of the direct method-based SLAM systems. For example, Zhu et al. [24] proposed a photometric transfer net (PTNet), which is trained to pixel-wisely remove brightness discrepancies between two frames without ruining the context information, to overcome the problem of brightness discrepancies. Liu et al. [25] proposed an enhanced visual SLAM algorithm based on the sparse direct method to solve the illumination sensitivity problem. Sheng et al. [26] filtered out the dynamic objects based on the semantic information to improve the positioning accuracy and robustness of DSO [21]. Zhou et al. [27] jointly optimized the 3D lines, points, and poses within a sliding window to consider the collinear constraint among the points to improve the robustness of the direct method.

The works introduced above can improve the robustness of the direct method to some extent. However, the research focusing on the influence of different camera imaging disturbances and semistatic objects is relatively lacking. During the long-term operation of the monocular SLAM system, the image quality of the camera will be affected by different disturbances from the external environment and internal sensors. In this paper, two main types of imaging disturbances are studied, namely, different noise on the camera and the brightness influence on the imaging process. The main noises on the camera include Gaussian noise and Salt-and-Pepper noise. Gaussian noise is often caused by the high temperature of the camera sensor running for a long time and mutual interference of internal circuit components [28]. Salt-and-Pepper noise is often caused by the faulty of the camera sensor, the wear of the camera lens, and the adsorption of dust in the air [29, 30]. The brightness influence on the imaging is a very common problem of the vision-based SLAM. For example, the accumulated irradiance exceeding the camera's dynamic range can cause the camera overexposure interference when the ambient brightness is not uniform [31, 32]. Another important influence on the robustness of the direct methods in the vision-based SLAM is the semistatic objects, which refer to objects that are static most of the time but will change at a certain moment, such as the cars parked on the side of the road. Semistatic objects are not suitable for being directly filtered out like dynamic objects because most of them are rich in texture and are suitable for estimating pose when they are static [33]. Thus, the main motivation of this paper is to study how to improve the robustness of the direct method-based SLAM system in different camera imaging disturbances and reduce the specific gravity of semistatic objects.

The main contributions of this paper are as follows: (1) A regional pixel information fusion method based on multiple average calculations is proposed to improve the robustness of the direct sparse odometry with loop closure- (LDSO-) based SLAM. (2) A side window strategy is introduced into the framework of the LDSO-based SLAM to enhance the edge-preserving property. (3) A method based on semantic information is presented to reduce the effects of nonstatic objects on the LDSO-based SLAM. So there are three main improvements of the proposed method, namely, a regional pixel information fusion method for robustness, a side window strategy for edge preserving, and the semantic-based strategy for the nonstatic objects. Compared with the existing methods, the proposed method improves the robustness of the direct method-based SLAM against multiple camera imaging disturbances, including Gaussian noise, Salt-and-Pepper noise, and camera overexposure, rather than just against a single disturbance.

The rest of this paper is organized as follows.  Section 2 gives out an overview of the background. The proposed algorithm is presented in Section 3. In Section 4, detailed quantitative and qualitative experimental results are provided. The discussions of the proposed algorithm are carried out in Section 5. Finally, Section 6 concludes this paper and gives out the future work.

## 2. Background

Direct method-based SLAM systems jointly estimate the position and posture changes of the camera by minimizing the photometric error in the image alignment. It makes direct methods more accurate and robust than feature-based methods in scenes that lack texture or are full of repetitive textures. However, the monocular direct methods suffer from the accumulated drift of global translation, rotation, and scale without closed-loop detection. This leads to inaccurate long-term trajectory estimation and mapping. In this paper, Direct Sparse Odometry with Loop closure (LDSO) [34] is focused on, which adds closed-loop detection to DSO for global optimization. The main process of LDSO is reviewed in this section.

### 2.1. Framework of LDSO

The algorithm framework of LDSO is shown in Figure 1. When a new frame of image is acquired, all the active 3D points in the current sliding window of the local bundle adjustment module are projected into this frame. The initial pose of this frame is estimated by direct image alignment. This frame is added to the local windowed bundle adjustment if it is judged as a new keyframe. Old or redundant keyframes and points are marginalized. The active keyframes and the marginalized keyframes rely on bag-of-words (BoW) for closed-loop detection and verification. If the closed-loop candidate is verified, it is added to the global pose graph for optimization.

### 2.2. Local Bundle Adjustment

In the local bundle adjustment module based on sliding window, 5–7 keyframes are maintained. Their parameters are jointly optimized by minimizing the photometric error. The photometric error is defined as

(1) $$\begin{array}{c} \min\sum_{T_{i},T_{j},p_{k}\in W}E_{i,j,k}, \end{array}$$

where *W* = {**T**_1_,…, **T**_*m*_, **p**_1_,…, **p**_*n*_} is the *m* keyframe poses represented as Euclidean transformation and *n* points of inverse depth parameterization in the sliding window. *E*_*i*,*j*,*k*_ is calculated by

(2) $$\begin{array}{c} E_{i,j,k}=\sum_{p\in N_{p_{k}}}w_{p}{\left\|\left(I_{j}\left[p^{\prime }\right]-b_{j}\right)-\frac{t_{j}e^{a_{j}}}{t_{i}e^{a_{i}}}\left(I_{i}\left[p\right]-b_{i}\right)\right\|}_{\gamma }, \end{array}$$

where *N*_**p**_*k*__ denotes the neighborhood pattern of **p**_*k*_; *a* and *b* are the affine light transform parameters; *t* denotes the exposure time; *I* is an image; *w*_**p**_ is a heuristic weighting factor; ‖·‖_*γ*_ is the Huber norm; and **p**′ denotes the reprojected pixel of **p** on *I*_*j*_, which is calculated by

(3) $$\begin{array}{c} p^{\prime }=\prod \left(R\Pi^{-1}\left(p,d_{p_{k}}\right)+t\right), \end{array}$$

where Π is the projection function from ℝ^3^ to Ω; **R** and **t** are the relative rotation and translation between the two frames; and *d*_**p**_ is the inverse depth of point **p**.

### 2.3. Closed-Loop Detection and Verification

In the LDSO SLAM, the DSO's point selection strategy has been modified to be more sensitive to corner points. The selected corner points are calculated as their ORB descriptors and packed into BoW. When the ORB descriptor of each keyframe is calculated, the closed-loop candidates of the keyframe are proposed by querying the BoW database. The similarity transformation from the closed-loop candidate to the current keyframe **S**_*cr*_ is optimized by minimizing 3D and 2D geometric constraints:

(4) $$\begin{array}{c} E_{loop}=\sum_{q_{i}\in Q_{1}}w_{1}{\left\|S_{cr}\Pi^{-1}\left(p_{i},d_{p_{i}}\right)-\Pi^{-1}\left(q_{i},d_{q_{i}}\right)\right\|}_{2}+\sum_{q_{j}\in Q_{2}}w_{2}{\left\|\prod \left(S_{cr}\Pi^{-1}\left(p_{j},d_{p_{j}}\right)\right)-q_{j}\right\|}_{2}, \end{array}$$

where *Q*_1_ and *Q*_2_ are the matched features in the current keyframe without and with depth, respectively; **p**_*i*_ denotes the reconstructed feature in the closed-loop candidates; *d*_**q**_ is the inverse depth of the feature **q**; and *w*_1_ and *w*_2_ are the weights to balance the different measurement units.

It can be noticed from equation (2) that the pose estimation of LDSO relies on minimizing the photometric error of the selected points. If the selected points are disturbed by imaging disturbances, equation (2) is converted into

(5) $$\begin{array}{c} E_{i,j,k}=\sum_{p\in N_{p_{k}}}w_{p}{\left\|\left(I_{j}\left[p^{\prime }\right]-b_{j}\right)-\frac{t_{j}e^{a_{j}}}{t_{i}e^{a_{i}}}\left(I_{i}\left[p\right]-b_{i}\right)\right\|}_{\gamma }+E_{n}, \end{array}$$

where *E*_*n*_ is the error due to imaging disturbances. As the intensity of the camera imaging disturbance increases, the optimization direction for minimizing the photometric error is more inclined to the error caused by the imaging disturbances rather than the estimated pose. Therefore, the robustness of LDSO in camera imaging disturbances is not strong enough.

## 3. Proposed Method

To enhance the robustness of the direct SLAM method, the points are fused with the surrounding pixels' information. The overview of the proposed method for obtaining and using fusion points is shown in Figure 2.

As shown in Figure 2, the area around each pixel is divided into blocks according to the side window strategy when a new frame arrives. The area block that crosses the image's edge the fewest times is chosen. This region block's pixel information is averaged into a single point. Multilayers of such pixel information fusion are superimposed to form a convolutional neural network (CNN) like structure [35, 36]. In the middle layer, semistatic objects are detected. The radiuses of the side window of the pixels belonging to the semistatic objects are increased in the back layers. The fusion points form the fused image. The points with sufficient gradient intensity and corners are selected using a dynamic grid search. These points are used in direct SLAM to improve the robustness of the system. The details of the proposed method are introduced as follows. The regional pixel information fusion is realized by multilayer fusion with a CNN-like structure. Then, the side window strategy is added to the fusion method for edge preservation. Finally, the radius of the side window is adjusted based on semantic information to reduce the weights of the semistatic objects.

### 3.1. Regional Pixel Information Fusion Method

As we know, the main reason why the robustness of feature-based SLAM is better than that of direct SLAM is that the feature carries the general information of pixels in a local area instead of a single pixel [37]. Therefore, to improve the robustness of LDSO in different camera imaging disturbances, a regional pixel information fusion method is introduced into the LDSO algorithm. Namely, each pixel can fuse the information of surrounding pixels, and the fusion intensity decreases as the distance between the pixels increases.

The mean filter is one of the most common methods of fusing pixels. Unlike other filters such as the median, max, and min filters, which select one pixel and discard others, the mean filter considers information from all pixels. In addition, the mean filter is simple to implement. So, a 3 × 3 mean filter is used to fuse eight neighborhood pixels into one pixel in this study. At the same time, referring to the characteristics of the classic convolutional neural networks (CNN) [38], the mean filters are stacked in the structure of CNN. In CNN, the stacked convolutional layers are considered to extract high-level features of the image so that these feature points can be used for object classification operations. Each feature point obtained contains information about a local area. The CNN-like structure of the multilayer fusion used in this study is shown in Figure 2.

**Remark 1 .**

The main reason for using the 3 × 3 mean filter in this paper is that it is the minimum size that can cover eight neighborhood information. Using the stacking structure, the 3 × 3 receptive field can be easily expanded to 5 × 5, 7 × 7, and other larger receptive fields. By this stacking structure, the closer the points in this area are to the edge, the fewer times they are repeatedly used and the less they affect the obtained feature points. These characteristics are precisely in line with our needs for fusing regional pixel information.

### 3.2. Side Window Strategy for Pixel Fusion Area Selection

The consistent use of the square area as the pixel fusion range can conveniently improve the overall robustness of the visual odometry, but it will also cause a certain degree of damage to the edges of the image. The more the layers are stacked, the greater the degree of damage. In image processing, this is called nonedge preservation [39]. As mentioned earlier, the points/features selected by LDSO are pixels with sufficient intensity gradients and corner features. Pixel fusion across the edges will reduce the gradient intensity of the pixels and blur the corner features. Since it makes the selected points difficult to gather at the edge, the point cloud map constructed is very unclear. Since the corner features are blurred and difficult to be extracted, it is difficult for LDSO to detect the closed-loop effectively.

To solve the above problems caused by the nonedge preservation of pixel fusion in the fixed square area, the side window strategy is introduced into LDSO [40]. The side window strategy treats each pixel as a potential edge point. Unlike the traditional pixel fusion method that takes the pixel's position as the center of the filter window, the side window strategy aligns the edge of the filter window with the pixel. Different from nonlinear anisotropic weightings such as the spatial weighting and gray value weighting of bilateral filters, which only reduce the diffusion of pixels along the edge normal direction, the side window strategy can cut off all the normal diffusion [41].

The details of the side window strategy proposed in our multilayer fusion are as follows:

1. Each pixel and its surroundings are divided into eight side windows, as shown in Figure 2. They are the side windows in eight directions: up (*U*), down (*D*), left (*L*), right (*R*), northwest (NW), northeast (NE), southwest (SW), and southeast (SE). The center point *p*_*i*_ of the pixel fusion is located on the side or corner of the window. The radius *r* of the side window determines the range of the pixel fusion.
2. The average value of the pixels in each side window is calculated as the output *q*_*n*_ of the side window, where *n* ∈ {*U*, *D*, *L*, *R*, NW, NE, SW, SE}.
3. Compare the distance measured by *L*_1_ norm between the output *q*_*n*_ of the eight side windows and the center point *p*_*i*_. The fusion output *p*^fusion^ of the center point *p*_*i*_ and its surrounding pixels is *p*^fusion^=*q*_*s*_, where

(6) $$\begin{array}{c} s=\underset{n\in \left\{U,D,L,R,NW,NE,SW,\text{SE}\right\}}{\arg\;\min}\left\{\left|q_{n}-p_{i}\right|\right\}. \end{array}$$

**Remark 2 .**

In the proposed multilayer superimposed pixel fusion strategy, the diffusion of pixels along the normal edge direction will be further amplified. And the side window strategy cuts off the possibility of pixels spreading along the normal direction of the edge, which is more suitable for our multilayer fusion.

The pseudocode of the proposed side window-based multilayer fusion method is summarized in Algorithm 1.

### 3.3. Semantic-Based Variable Radius Side Window Strategy

When humans use their eyes to estimate their position and remember the environment, they do not take all the objects they see into consideration. Instead, they focus on static objects such as walls and pillars and use semistatic objects that are stationary most of the time, such as cars parked on the side of the road, as a reference. Inspired by this, a semantic-based variable radius side window strategy is proposed to assign weights to static and semistatic objects.

First, in the first half of the stacked structure of pixel fusion, a smaller radius for the side window is used. In multilayer pixel fusion, due to the smaller coverage area, the side window with a smaller radius can make the image retain more details such as edges while reducing the impact of camera imaging disturbances. Subsequent object detection in a camera imaging disturbed environment is carried out on this basis.

Second, Yolov5 (one of the popular object detection deep networks) is used to distinguish static and semistatic objects in the input images. Yolov5 is the latest version of the Yolo object detection algorithm [42, 43]. The main reason for using the Yolov5 network is that Yolov5 can also maintain a higher processing frame rate under lower hardware conditions while achieving the accuracy of the current state-of-the-art technology. In this study, the pretrained Yolov5 model on the Microsoft COCO (Common Objects in Context) dataset is used to extract object location and category semantic information [44]. Common movable categories such as bicycles, cars, motorcycles, buses, and trucks in the COCO dataset are marked as semistatic objects.

Third, in the second half of the stacked structure of the pixel fusion, a slightly larger radius is used for the side windows of the regions where the semistatic objects are detected. A side window with a larger radius is more likely to contain more image edges. The selection principle of the side window is to select the side window whose output is most similar to the center pixel. The larger the edge gradient of the image within the coverage of the side window, the more dissimilar the output is from the center pixel. Therefore, the side window strategy is more inclined to retain the image edges with large gradients. Edges with smaller gradients in the side window will be blurred. With repeated pixel fusion, the obvious image edges in the semistatic object area will be preserved, while the pixel gradients inside will be reduced.

**Remark 3 .**

The specific gravity of the point in the semistatic object area selected by the LDSO with a high gradient intensity will decrease. The preserved obvious image edges can provide enough corner features for LDSO. In this way, a static object-based and semistatic object-assisted approach similar to the human positioning strategy is achieved.

A summary of the proposed points selection strategy based on the side window with semantic-based variable radius is given in Algorithm 2.

Overall, the workflow of the proposed variable radius side window direct SLAM method is summarized as follows:

**Step 1 .**

The radius parameters applicable to different regions are selected based on semantic information.

**Step 2 .**

The different radius parameters are applied to the side window strategy to form a variable radius side window strategy.

**Step 3 .**

The semantic information-based variable radius side window strategy is applied to a multilayer stacked pixel blender to fuse regional pixel information.

**Step 4 .**

The points are selected according to Algorithm 2 on the points fused with local information.

**Step 5 .**

The selected points are used to estimate the camera pose by minimizing equation (2) and perform global optimization by minimizing equation (4) when loop closures are detected.

## 4. Experimental Results and Analysis

In this section, the proposed method is comprehensively evaluated on outdoor datasets (KITTI dataset) and indoor datasets (TUM RGB-D dataset), which are introduced as follows:

1. KITTI dataset [45, 46]: this dataset is currently the most extensive dataset in the world for evaluating computer vision algorithms in autonomous driving scenarios. It contains real image data collected in outdoor scenes such as urban areas, villages, and highways. The “00–10” sequences in this dataset provide ground truth, which are used in this study.
2. TUM RGB-D dataset [47, 48]: this dataset provides RGB-D data and ground-truth data intending to establish a novel benchmark for the evaluation of visual odometry and visual SLAM systems. In this paper, the sequences “freiburg1_xyz,” “freiburg2_xyz,” “freiburg2_rpy,” “freiburg1_desk,” and “freiburg1_desk2” are selected, which were all acquired in the office interior scene with rich texture.

The main reason for using the two datasets is that both of them provide ground truth, which is required for the quantitative evaluation. Because there is a certain natural camera overexposure problem in the two datasets [49], they are used directly to test the proposed method under the disturbance of camera overexposure. In addition, Gaussian noise and Salt-and-Pepper noise are added to the two datasets in these experiments to further test the proposed method under different camera sensor noises. In this paper, the variance of Gaussian noise added is 0.003, and the rate of Salt-and-Pepper noise added is 10%. The noise addition operation and the noise-adding parameters in this study are relatively common in the literature [50, 51].  Figure 3 shows an example scene before and after adding two kinds of noise.

### 4.1. Quantitative Evaluation

In this study, the proposed method is based on the side window fusion strategy on the direct method-based SLAM. Here, it is compared with the general direct sparse odometry method (DSO) and the general direct sparse odometry with loop closure (LDSO). In this paper, the large-scale direct monocular SLAM (LSD-SLAM) is not compared because its tracking robustness is not as good as DSO [52]. To further discuss the performance of our method, ORB-SLAM3 is also added for comparison, which is one of the state-of-the-art methods based on the feature-based method [53, 54]. The root mean squared error of absolute trajectory error (RMSE_ATE_) is used to evaluate the performance of these methods [55].

#### 4.1.1. On the KITTI Dataset

Firstly, some comparison experiments are conducted on the KITTI dataset to show the robustness of the proposed method in the face of different camera imaging disturbances. The results with no noise added, Gaussian noise, and Salt-and-Pepper noise are listed in Tables 1–3, respectively. The missing values in the tables mean tracking failures.

The results in Table 1 show that our method can achieve similar or better performance compared with the other direct methods in the sequences without added noise. The results on the sequences without added noise show that the performance of the proposed method is obviously better than the general LDSO method on the sequences “KITTI_00” and “KITTI_02,” where the RMSE values of the proposed method are 32.42% and 51.91% less than the general LDSO method. The main reason is that the sequences “KITTI_00” and “KITTI_02” have a large number of scenes in the shade of trees (see Figures 4(a) and 4(c)), and frequent changes in ambient light bring more frequent camera overexposure problems to the images. The results show that the proposed method can deal with the camera overexposure interference on the direct methods effectively.

In the sequences with Gaussian noise, we can see that the performance of the general direct methods decreases obviously on all of the sequences in the KITTI dataset, but the proposed method is not seriously affected by the Gaussian noise (see Table 2). In particular, the other direct methods fail to track in sequence “KITTI_03,” “KITTI_04,” and “KITTI_09” while our method still works. The results in Table 2 show that the proposed method outperforms the general LDSO method by more than 13.7% on all of the sequences in the KITTI dataset. In the sequences with Salt-and-Pepper noise, DSO and LDSO are entirely inoperable, while our method obtains good performance (see Table 3).

Compared with ORB-SLAM3, our method obtains slightly better performance on the sequences without added noise, except sequences “KITTI_08,” “KITTI_09,” and “KITTI_10.” The main reason is that these sequences contain very rich textures that are more suitable for feature-based methods. In particular, ORB-SLAM3 will track failure in the sequence “KITTI_01,” whether the noise is added or not. This is due to the fact that the sequence “KITTI_01” is a very texture-deficient highway scene and is not suitable for feature-based SLAM methods (see Figure 4(b)).

Although ORB-SLAM3 performs better in the face of Gaussian noise (see Table 2), ORB-SLAM3 is unavailable under the influence of Salt-and-Pepper noise (see Table 3). By contrast, the results show that our method performs more consistently in different camera imaging disturbances than other methods (see Tables 2 and 3).

To compare the robustness in different camera imaging disturbances more clearly, the absolute pose errors (APE) with respect to translation on the example sequence “KITTI_07” in different noises are shown in Figure 5. Here, the main reason for using the sequence “KITTI_07” as the example is that this sequence has a medium sequence length in the KITTI dataset. In the next part of this paper, the sequence “KITTI_07” is also used as the study object, where the reason is not further explained. The lack of the APE curves of DSO and LDSO in the sequence with Salt-and-Pepper noise is due to their inability to work. Notice that our method has more consistent APE curves in different noises, and all the APEs of our method are less than 5.0%. This experiment highlights that our strategy effectively improves the robustness of direct SLAM when facing different camera imaging disturbances outdoors.

#### 4.1.2. On the TUM RGB-D Dataset

Secondly, some experiments are conducted on the TUM RGB-D dataset to verify whether our strategy has the effect of improving robustness in indoor environments. Since DSO and LDSO perform very similarly in this case, our method is only compared with LDSO. In this dataset, there are many blurred images with smears, as shown in Figure 6. In this experiment, because the selected sequences are relatively short, the difference in RMSE is not apparent. Thus, we mainly compare whether the tracking of the SLAM system based on different methods is successful. The results are shown in Tables 4–6.

The results in this experiment show that the SLAM system will fail easily after adding noise to the images. Note that, in the sequences in which no noise is added, both our method and LDSO can track successfully (see Table 4). After adding different noises to the sequences, LDSO becomes more prone to failure tracking, while our method still tracks successfully (see Tables 5 and 6). This experiment highlights that our approach can still improve the robustness of direct SLAM under different camera imaging disturbances when faced with a poor indoor image input.

### 4.2. Qualitative Evaluation

This section mainly conducts a qualitative evaluation of the completeness and the clarity of the predicted trajectory map and the constructed point cloud map in the camera imaging disturbances. Examples of the point cloud map constructed on the sequence “KITTI_07” are shown in Figure 7. The results show that our method is similar to LDSO in the absence of noise interference. When disturbed by Gaussian noise and Salt-and-Pepper noise, LDSO is negatively affected to varying degrees, while our method has a better and more stable performance in the trajectory prediction and point cloud map construction. The main reason is that our method uses the multilayer pixel fusion features based on the side window strategy instead of directly using the original pixels, which can improve the robustness of the direct method-based SLAM in different camera imaging disturbances.

## 5. Discussion

The total performances of the proposed method have been proved on different datasets by some comparison experiments in Section 4. In this section, some additional comparison experiments are conducted to discuss the performance of our method in different intensities of camera imaging disturbances. In addition, the performance of the key improvement of the proposed method, namely, the points selection strategy, is further discussed. At last, the proposed method is tested in real-world applications to demonstrate the effectiveness of the proposed method.

### 5.1. Performance in Camera Imaging Disturbances of Different Intensities

Firstly, the performance of our method in the camera imaging disturbances of different intensities is discussed, where some expanded comparison experiments are conducted under the sensor noise of different intensities and the camera overexposure with different frequencies.

#### 5.1.1. About Different Noise Intensities

The performance of our method in the camera sensor noise of different intensities is discussed on the sequence “KITTI_07.” The comparison experiments are carried out separately in Gaussian noise and Salt-and-Pepper noise with different intensities. The variance of Gaussian noise ranges from 0.001 to 0.009 and is incremented by a step size of 0.002. The rate of Salt-and-Pepper noise added ranges from 2% to 10%, and the step size is 2%. The results are shown in Tables 7 and 8. For Gaussian noise, DSO tracking fails when the variance is greater than 0.005. LDSO tracking fails when the variance is greater than 0.003. Our method tracks successfully at all noise intensities and performs stably when the variance is below 0.005. This reflects that our method is more robust than other direct methods in different intensities of Gaussian noise. For Salt-and-Pepper noise, both DSO and LDSO fail to track when the noise addition rate is greater than 2%. Our method can track successfully and perform stably at all noise addition rates. It can be seen that our method is more robust than other direct methods in different intensities of Salt-and-Pepper noise. ORB-SLAM3 can also track successfully in all intensities of Gaussian noise and performs stably when the variance is below 0.007. While ORB-SLAM3 outperforms our method in robustness under different intensities of Gaussian noise, it fails to track at all addition rates of Salt-and-Pepper noise.

#### 5.1.2. About Different Overexposure Frequencies

To discuss the performance of our method under the interference of camera overexposure, the sequence “KITTI_01,” which suffers little from camera overexposure, is experimented with adding simulated camera overexposure disturbance at different frequencies. The camera overexposure addition operation in this study is similar to other pieces of literature [56]. The number of interval frames at which overexposure interference is added ranges from 30 to 10 and is decreased by a step size of 5. The results are shown in Table 9.

The results in Table 9 show that our method performs close to LDSO when the camera overexposure interference is not very serious. However, when the overexposure interference interval is 20 frames, the proposed method outperforms the general LDSO method by more than 46%. In addition, LDSO starts to fail to track when the overexposure interference interval is lower than 15 frames, while our method can still work when the overexposure interference interval is bigger than 10 frames. ORB-SLAM3 fails to track in the sequence “KITTI_01” under the added camera overexposure interference. The results of this experiment show that the proposed method has better performance under the camera overexposure interference.

### 5.2. About Points Selection Strategy

Secondly, the effect of the points selection strategy of our method to improve the robustness of direct method-based SLAM is discussed.  Figure 8 shows the selection of points in an example scene with different types of noise. Here, our points selection strategy is compared with that of the general LDSO. It is easy to notice that the points selected by our strategy are more consistent in different noises. It is not easy for LDSO to detect closed loops under the influence of Gaussian noise. Gaussian noise creates texture in untextured areas. These textures are selected as the basis for closed-loop detection, which easily leads to the failure of closed-loop detection. In Salt-and-Pepper noise, LDSO is entirely inoperable. The reason is that the image-gradient-based features selected by LDSO are easily located at the position of the Salt-and-Pepper noise (see Figure 8(c)). These randomly generated noise positions cannot be used as the basis for estimating camera pose. As shown in Figure 8(a), the points selected by our method are significantly less than that by LDSO and are mainly distributed on the apparent edges of the semistatic objects such as cars parked on the side of the road. The consistent selection of points of our method improves the robustness of direct method-based SLAM.

The comparison results of RMSE_ATE_ based on the proposed semantic-based variable radius side window (SVR-SW) and the fixed radius side window in the general LDSO (FR-SW) are shown in Table 10. Here, the sequences “07” and “08” of the KITTI dataset are used, which contain more semistatic objects. It can be noticed that the proposed SVR-SW strategy achieves better performance on different noises. The main reason is that the semantic-based variable radius side window can reduce the weight of selected points of semistatic objects to improve the performance of direct method-based SLAM in scenes with more semistatic objects.

### 5.3. Experiment in Real Scene

Thirdly, to discuss the performance of our method in real scenes, an experiment is conducted on a real-world dataset collected outdoors by the Zenmuse X5S camera mounted on the DJI Inspire 2 drone [57]. In reality, the camera imaging disturbances often do not exist all the time but are sudden and random. For simulation of this situation, Gaussian noise and Salt-and-Pepper noise are artificially added to parts of this dataset. Some images added with noise are shown in Figure 9, which have obvious brightness changes due to the shade of trees and lots of semistatic objects in the real scene, such as bicycles and cars. The real-world dataset is collected along the road to easily judge whether our method estimates the correct trajectory using the satellite map. The experimental result of this self-collected real dataset is shown in Figure 10. It can be seen that the trajectory estimated by our method does not deviate from the road due to the camera imaging disturbances, including the artificially added noise and the natural brightness changes. Our method performs good robustness on different camera imaging disturbances in real scenes.

## 6. Conclusion

The robustness in the camera imaging disturbances of the direct method-based SLAM is studied in this paper, and a concept of side windows is introduced into this visual SLAM system. Based on this concept, a multilayer stacked pixel blender is used to process the input images, which can significantly reduce the blurring effects on the edges of the images. In addition, the size of the fusion window can be adjusted based on semantic information to reduce the proportion of selected points on semistatic objects. At last, to more clearly evaluate the robustness of the proposed method under different camera imaging disturbances, the public datasets enhanced with different camera imaging disturbances are used to perform detailed quantitative and qualitative experiments. The results demonstrate that our strategy can improve the robustness of the direct method-based SLAM against the different camera imaging disturbances, including various sensor noises and camera overexposure. Furthermore, the results of the real-world experiment show that the proposed method can work efficiently in real-world applications. In the future, how to further improve the robustness of the visual SLAM method while improving efficiency by using different fusion methods should be studied, such as deep neural networks.

## Figures and Tables

**Figure 1:** The framework of the LDSO method.

**Figure 2:** The overview of the proposed method for obtaining and using fusion points.

**Figure 3:** Comparison of the example scene before and after adding noise. (a) The original image. (b) The image after adding Gaussian noise. (c) The image after adding Salt-and-Pepper noise. Note that the effect of the added noise is noticeable.

**Figure 4:** Example scenes for sequences “KITTI_00,” “KITTI_01,” and “KITTI_02” in the KITTI dataset: (a) is from the sequence “KITTI_00”; (b) is from the sequence “KITTI_01”; (c) is from the sequence “KITTI_02.” The sequences “KITTI_00” and “KITTI_02” are the sequences with more camera overexposure interference, while “KITTI_01” is the sequence with little camera overexposure interference.

**Figure 5:** Comparison of APE with respect to translation in different noises on the sequence “KITTI_07”: (a) APE of DSO. (b) APE of LDSO. (c) APE of our method. Note that the performance gap of our method is significantly smaller than that of DSO and LDSO. In particular, DSO and LDSO do not work in the sequence with Salt-and-Pepper noise, and the results in this case cannot be added for comparison. Besides, the performance of our method is better than the others overall.

**Figure 6:** Blurred image with smears in TUM RGB-D dataset.

**Figure 7:** Sample outputs of the sequence “KITTI_07”: (a), (b), and (c) are the outputs on the sequence with no added noise, Gaussian noise, and Salt-and-Pepper noise, respectively. Left: LDSO's outputs. Right: our method's outputs. Note that, in the sequence without adding noise, the quality of our method's trajectory estimation and point cloud map construction is similar to that of LDSO. In the sequence with Gaussian noise added to LDSO, the closed-loop cannot be detected, and the trajectory estimation in the second half is wrong. LDSO does not work in the sequence with Salt-and-Pepper noise added. Our strategy achieves a more robust performance under different noise interferences.

**Figure 8:** Point selection results of our strategy and LDSO in different noises: (a), (b), and (c) are the images from the KITTI dataset with no added noise, Gaussian noise, and Salt-and-Pepper noise, respectively. Top rows: point selection results of LDSO. Bottom rows: point selection results of our strategy. Note that the points selected by our strategy are more consistent in different noises. Moreover, on semistatic objects such as cars parked on the side of the road, the points selected by our approach are significantly less than those by LDSO and are mainly distributed on the apparent edges.

**Figure 9:** Some images in the real scene added with noise. (a) Added with Gaussian noise. (b) Added with Salt-and-Pepper noise.

**Figure 10:** Result of experiment in real scene. (a) The trajectory estimated by our method, which is marked with a yellow curve. (b) The approximate trajectory on the satellite map, which is marked with a red dashed line.

**Algorithm 1:** Side window-based multilayer fusion.

**Algorithm 2:** Semantic variable radius side window-based points selection.

**Table 1:** RMSE_ATE_ on KITTI dataset with no noise added.

Method	No noise added											
	KITTI_00	KITTI_01	KITTI_02	KITTI_03	KITTI_04	KITTI_05	KITTI_06	KITTI_07	KITTI_08	KITTI_09	KITTI_10	Average
DSO [21]	115.035	31.811	152.463	2.030	0.755	49.981	54.004	17.576	114.391	70.534	14.661	56.658
LDSO [34]	7.360	9.972	47.245	2.342	0.800	4.166	12.805	1.691	114.739	69.803	14.815	25.976
ORB-SLAM3 [54]	9.265	—	22.025	2.117	1.223	4.034	16.196	1.688	38.114	7.243	7.771	10.968
Ours	4.974	9.710	22.722	2.183	0.857	3.540	12.798	1.789	99.579	52.469	14.210	20.439

*Note.* “—“ means tracking failure. The average value is calculated based on the number of successes.

**Table 2:** RMSE_ATE_ on KITTI dataset with Gaussian noise.

Method	Gaussian noise											
	KITTI_00	KITTI_01	KITTI_02	KITTI_03	KITTI_04	KITTI_05	KITTI_06	KITTI_07	KITTI_08	KITTI_09	KITTI_10	Average
DSO [21]	115.771	56.143	185.187	—	—	50.185	59.382	38.812	127.674	—	15.287	81.055
LDSO [34]	22.543	23.052	169.247	—	—	44.010	58.729	53.481	130.993	—	16.277	64.792
ORB-SLAM3 [54]	10.645	—	59.868	2.860	1.911	9.250	19.249	1.932	42.931	8.223	8.776	16.565
Ours	17.772	13.023	120.380	2.133	1.093	5.740	13.491	1.973	102.206	52.664	14.042	31.320

*Note.* “—“ means tracking failure. The average value is calculated based on the number of successes.

**Table 3:** RMSE_ATE_ on KITTI dataset with Salt-and-Pepper noise.

Method	Salt-and-Pepper noise											
	KITTI_00	KITTI_01	KITTI_02	KITTI_03	KITTI_04	KITTI_05	KITTI_06	KITTI_07	KITTI_08	KITTI_09	KITTI_10	Average
DSO [21]	—	—	—	—	—	—	—	—	—	—	—	—
LDSO [34]	—	—	—	—	—	—	—	—	—	—	—	—
ORB-SLAM3 [54]	—	—	—	—	—	—	—	—	—	—	—	—
Ours	19.798	10.464	108.448	2.252	0.806	11.581	12.463	2.238	101.590	52.177	14.937	30.614

*Note.* “—“ means tracking failure.

**Table 4:** RMSE_ATE_ on TUM RGB-D dataset with no noise added.

Method	No noise added				
	fr1_xyz	fr2_xyz	fr2_rpy	fr1_desk	fr1_desk2
LDSO [34]	0.061	0.011	0.046	0.774	0.904
Ours	0.063	0.012	0.043	0.780	0.905

**Table 5:** RMSE_ATE_ on TUM RGB-D dataset with Gaussian noise.

Method	Gaussian noise				
	fr1_xyz	fr2_xyz	fr2_rpy	fr1_desk	fr1_desk2
LDSO [34]	—	0.096	—	0.518	—
Ours	0.156	0.010	0.060	0.801	0.756

*Note.* “—” means tracking failure.

**Table 6:** RMSE_ATE_ on TUM RGB-D dataset with Salt-and-Pepper noise.

Method	Salt-and-Pepper noise				
	fr1_xyz	fr2_xyz	fr2_rpy	fr1_desk	fr1_desk2
LDSO [34]	—	—	—	0.841	—
Ours	0.129	0.011	0.058	0.796	0.871

*Note.* “—” means tracking failure.

**Table 7:** RMSE_ATE_ comparison in Gaussian noise of different intensities.

Variance	DSO [21]	LDSO [34]	ORB-SLAM3 [54]	Ours
0.001	24.396	2.504	1.872	1.655
0.003	38.812	53.481	1.932	1.973
0.005	45.968	—	2.101	2.946
0.007	—	—	2.566	12.343
0.009	—	—	10.242	13.816

*Note.* “—” means tracking failure.

**Table 8:** RMSE_ATE_ comparison in Salt-and-Pepper noise of different intensities.

Addition rate (%)	DSO [21]	LDSO [34]	ORB-SLAM3 [54]	Ours
2	35.500	35.525	—	1.409
4	—	—	—	1.602
6	—	—	—	1.755
8	—	—	—	2.225
10	—	—	—	2.238

*Note.* “—” means tracking failure.

**Table 9:** RMSE_ATE_ comparison under interference of camera overexposure at different frequencies.

Interval frames	DSO [21]	LDSO [34]	ORB-SLAM3 [54]	Ours
30	32.946	11.866	—	11.522
25	34.257	12.248	—	11.836
20	—	22.240	—	11.885
15	—	—	—	13.333
10	—	—	—	—

*Note.* “—” means tracking failure.

**Table 10:** RMSE_ATE_ comparison of whether using semantic-based variable radius side window.

Method	No noise added		Gaussian noise		Salt-and-Pepper noise	
	KITTI_07	KITTI_08	KITTI_07	KITTI_08	KITTI_07	KITTI_08
FR-SW	2.256	106.652	2.794	112.754	2.471	106.093
SVR-SW	1.789	99.579	1.973	102.206	2.238	101.590

## Data Availability

Publicly available datasets were analyzed in this study. These data can be found at http://www.cvlibs.net/datasets/kitti/eval_odometry.php and https://vision.in.tum.de/data/datasets/rgbd-dataset/download.
